# Effects of Smartphone Overdependence and the Quality of Friendship on Depression among High School Students

**DOI:** 10.1155/2022/3932326

**Published:** 2022-05-21

**Authors:** Son Sung-min, Jeon Byoung-jin

**Affiliations:** ^1^BK21FOUR R&E Center for Learning Health Systems, Korea University, Seoul, Republic of Korea; ^2^Department of Occupational Therapy, Kangwon National University, Samcheok, Republic of Korea

## Abstract

This study analyzes the effects of smartphone overdependence and the quality of friendship on depression among high school students in Korea. The study subjects were 121 high school students. Smartphone overdependence was assessed using the smartphone overdependence scale for adolescents, depression was assessed using the Korean version of the patient health questionnaire-9, and the quality of friendship was assessed using the friendship quality questionnaire. The results of the correlation analysis showed statistically significant differences among all the variables. The results of the multiple linear regression analysis showed that smartphone overdependence increases the depression level, whereas the quality of friendship lowers it. To decrease depression among high school students, smartphone overdependence and the quality of friendship should be managed appropriately. Moreover, the causal relationships and mediating effects between smartphone overdependence and the quality of friendship should be analyzed.

## 1. Introduction

The development of smartphones is playing a leading role in the changes as modern society enters the Fourth Industrial Revolution era. This development is accelerating worldwide, and the use of smartphones is also increasing rapidly [1]. According to the recent survey by a US research institute, South Korea has the highest penetration rate of smartphones globally [2]. Smartphones can increase the efficiency of work processes as well as be used as educational tools [3]. In addition, they allow people to form interpersonal relationships and maintain those relationships using social networking services. In particular, smartphones are important tools for individuals to form their own culture, express themselves, and decrease the stress of daily life [4].

However, despite their positive functions of smartphones, various social problems have been induced by dysfunctional smartphone use, and these problems have occurred in various age groups from children to adults [2]. Among these social problems, smartphone overdependence has increased significantly, with a concurrent rise in the number of studies examining this phenomenon [1]. Smartphone overdependence indicates the state in which an individual's ability to control their smartphone use is markedly decreased to the point that using a smartphone is considered to be the most important activity in their daily life [5]. In addition, it is defined as a state of the excessive use of smartphones despite experiencing negative consequences including a decrease in academic achievement and work efficiency [6].

The period of high school is a transitional period for individuals to prepare for adulthood. During this life stage, it is important to achieve one's core goals to form appropriate social roles and build interpersonal skills [7]. Kim et al. [8] reported that the high school period enables students to perform social roles by learning the appropriate attitudes and communication skills as a preliminary member of society. This stage also allows them to experience relationships with others as well as form self-confidence, emotional stability, and self-identity. However, physical, sexual, cognitive, and emotional changes occur rapidly in this period, which can create negative emotions such as uncertainty and disconnection [8]. Accordingly, high school students may lose their direction due to a lack of awareness of their existence and values, and failing to form the correct values and a sense of self-congestion leads to various problems [9].

In particular, if such problems affect the formation of friendship networks and their quality, conflicts in the performance of social roles may be induced; such problems in social interaction and adaptation may be caused by the inability to accept and respond to others [8]. Moreover, excessive demand to perform social roles can increase the psychological burden and stress of high school students, inducing physiological and psychological reactions and thus stress [9]. Further, these problems can induce depression, which is considered to be the most serious psychological problem in modern society and one that affects high school students' daily and school life. Depression, a typical psycho-emotional symptom that appears in daily life, is also a neuropsychological symptom that arises due to negative moods such as distress and lethargy and emotional problems caused by a decrease in activity performance [10].

Various studies have analyzed the level of smartphone overdependence of high school students. However, most have only reported problems related to their academic achievement [4, 11], adaptation to school life [12], and friendships [13]. Moreover, studies of the psychological problems caused by smartphone overdependence among high school students have only analyzed the outcomes of stress, self-efficacy, and self-control [14] as well as the effects on cyberbullying [15]. In addition, although studies have analyzed the link between depression and the quality of friendship, they are scarce, and no studies have thus far examined the relationship between depression and the quality of friendship based on smartphone overdependence.

Therefore, this study was performed to analyze the effects of smartphone overdependence and the quality of friendship on depression among high school students in Korea.

## 2. Materials and Methods

### 2.1. Study Subjects and Period

The study subjects were 121 high school students attending in the W high school in J city in Korea. Following Hwang et al. [1], they were sampled using convenience sampling. Included individuals were those who use a smartphone, have not been diagnosed with a learning disability or mental disorder or have no prior history of them, and agreed to participate in this study voluntarily. The participants were recruited from the school with the cooperation of their teacher at the beginning of the study. The purpose and content of this study were provided in an online form.

The number of study subjects was calculated using the G∗Power 3.1.9.4 software, with an effect size of .50, a significance level of .05, a power of.90, and a two-sided test [1]. As a result, at least 42 individuals were required as the subjects in this study. However, 121 high school students eventually participated. Consent was provided based on the ethical standards of the Declaration of Helsinki. Before participating, the subjects received a sufficient explanation of the purpose and methods of this study. Accordingly, this led to their voluntary decision to participate in this study. Written consent was provided online due to the social conditions caused by the COVID-19 pandemic. This study was conducted for eight weeks from April to June 2020.

### 2.2. Study Procedure

To analyze the effects of smartphone overdependence and the quality of friendship on depression, a single-group study design was applied, and a causal analysis of the variables was performed. Data collection and assessment were performed using an online survey considering the COVID-19 pandemic situation. Each assessment was conducted by an occupational therapist, who is an author of this paper. As noted above, before the online assessment, a sufficient explanation of the purpose and methods of this assessment and study was provided to the study subjects for them to understand. The assessment was conducted in a comfortable and stable condition with few distractions in the environment, which induced the participants to respond to the assessment items individually.

### 2.3. Smartphone Overdependence Assessment

The smartphone overdependence scale for adolescents was used to measure the level of smartphone overdependence among the study subjects. This integrated scale developed by the National Information Society Agency in Korea in 2016 is based on the standardized internet dependence scale and smartphone dependence scale developed in 2011. It is designed to measure the level of smartphone overdependence using a self-report 10-item questionnaire divided into three sub-areas: failure of accommodation, salience, and problematic outcome. Each score is measured on a four-point Likert scale from 1 to 4, and the total score ranges from 10 to 40 points. A higher score indicates a higher level of smartphone overdependence. Specifically, those scoring 31 points or more are classified as the high risk group, and those scoring 23 to 30 points are classified into the potential risk group. The Cronbach's *α* of the smartphone overdependence youth scale was .85 during development [6] and the Cronbach's *α* in this study was .86.

### 2.4. Depression Assessment

The Korean version of the Patient Health Questionnaire-9 (PHQ-9) was used to measure the level of depression among the study subjects. The PHQ-9 was translated into Korean and modified by Cho et al. [16]. This assessment aims to meet the diagnostic criteria for major depressive disorders in DSM-V. It is a self-report questionnaire that can sensitively identify depression. In addition, the PHQ-9 is a useful assessment in clinical settings because it has higher sensitivity and specificity than the SDS and BDI assessments used to measure depression [17]. The PHQ-9 consists of nine items, and each score is measured on a four-point Likert scale from 0 to 3. The total score of the PHQ-9 ranges from 0 to 27 points. A higher score indicates a higher level of depression. If the total score is 10 or more, it is classified as depression. The Cronbach's *α* of the PHQ-9 was .85 during development. When a score of 10 or more was judged as a cut-off point, sensitivity was reported to be 81.8 and specificity to be 89.9 [16]. The Cronbach's *α* in this study was.85.

### 2.5. Quality of Friendship Assessment

The Korean version of the friendship quality questionnaire (K-FQQ) was used to measure the quality of friendship among the study subjects. The K-FQQ was developed by Parker and Asher [18] and then modified by Kim for the Korean setting [19]. The K-FQQ consists of 21 items, including conflict resolution, help and guidance, company and entertainment, recognition and consideration, and close interaction. Each score is measured on a five-point Likert scale from 1 to 5, and the total score of the K-FQQ ranges from 21 to 105 points. A higher score indicates a higher quality of friendship. The Cronbach's *α* of the K-FQQ was .914 during development [20], and the Cronbach's *α* in this study was .957.

### 2.6. Statistical Analysis

The collected data for each question were coded and analyzed using STATA version 14.2. The general characteristics of the study subjects were analyzed using descriptive statistics, and the correlations among the variables were analyzed using correlation analysis. Moreover, to verify the causal relationships among the variables, in the regression analysis, White's test was performed to confirm homoscedasticity, and then multiple linear regression analysis using robust diagonally weighted least squares (RDWLS) was performed. The statistical significance level was set to 95%.

## 3. Results

### 3.1. General Characteristics of the Subjects

Table 1 shows the general characteristics of the study subjects. The 121 high school students had an average age of 16.69 years, and 70 were boys (57.85%). They were all in the second grade.

### 3.2. Results of the Analysis of each Variable

As shown in Table 2, for smartphone overdependence, the mean number of points was 20.36, and the range was 29 points from a minimum of 10 points to a maximum of 39 points. The skewness value was .225, and kurtosis was .045. For depression, the mean number of points was 4.22, and the range was 27 points from a minimum of 0 points to a maximum of 27 points. The skewness value was 2.275, and kurtosis was 6.591. For the quality of friendship, the mean number of points was 79.33, and the range was 44 points from a minimum of 61 points to a maximum of 105 points. The skewness value was .109, and kurtosis was -.186. The results of each variable were confirmed to satisfy the criteria for a normal distribution [21].

### 3.3. Results of the Correlation Analysis among the Variables

As shown in Table 3, there was a positive correlation between smartphone overdependence and depression (*r* = .343, *p* < .01) and a negative correlation between smartphone overdependence and the quality of friendship (*r* = −.203, *p* < .05). In addition, there was a negative correlation between depression and the quality of friendship (*r* = −.600, *p* < .01). Thus, these results confirmed that as the degree of smartphone overdependence increases, the level of depression increases and the quality of friendship decreases.

### 3.4. Results of the Multiple Linear Regression Analysis among the Variables

As heteroscedasticity was suspected (see Table 4), White's test was performed. The results in Table 5 show that homoscedasticity was rejected (*p* < .001), suggesting a high possibility of heteroscedasticity. To address these problems, multiple linear regression analysis with RDWLS was performed using STATA software.

Table 6 shows the results of the multiple linear regression analysis with RDWLS. The explanatory power of smartphone overdependence and the quality of friendship as the independent variables for the depression level of the study subjects was 41.1% (R^2^ = .411), and the research model was therefore confirmed to be suitable (F = 20.39, *p* < .001). In detail, smartphone overdependence had a positive effect on the depression level (Coef. = .203, *B* = .231, *p* < .05), whereas the quality of friendship had a negative effect (Coef. = −.2261, *B* = −.553, *p* < .001). According to these results, the higher the effect of the depression level on smartphone overdependence and the lower the quality of friendship, the higher the depression level.

## 4. Discussion

In this study, the results of the analysis showed the positive effect of smartphone overdependence on depression among high school students, indicating that if the level of smartphone overdependence increases, the depression level increases as well. Generally, high school students use their smartphones to escape from the psychological burden and stress of learning and social interaction as well as control their emotion and mood in daily and school life [12]. Students spend more time using their mobile phone than ever before, and they are comfortable using their smartphone to communicate. Hence, such use places them in a positive psychological situation and makes their life easier [22].

In addition to the clear communication benefits that smartphones provide, their high usability influences people's daily habits (e.g., sending text messages while walking) and encourages users, especially young people, to spend a lot of time on their smartphone daily [22–24]. In Korea, smartphone use by high school students is rapidly increasing and causing various social problems. According to the 2019 Youth Survey in Korea, four out of five high school students own a smartphone, and 29.3% of those aged 10–19 years are in the high-risk group of smartphone overdependence [25]. Moreover, high school students account for 28.3% of the high-risk group and are significantly more overdependent on smartphones than middle school students [26].

Smartphone-related risks have been investigated in terms of the various health conditions, with particular attention paid to the link between electromagnetic field exposure and headache, fatigue, and other non-specific symptoms [22, 27]. Shim et al. [28] reported that the use of smartphones increases time alone as well as smartphone dependence. In addition, from a neurophysiological point of view, they reported that visual stimulation from the smartphone causes functional problems in the frontal lobe of the cerebral cortex in the brain, increasing problems related to impulse control and thinking and judgment. Kim et al. [8] also reported that smartphone overdependence limits the cognitive processes of thinking and judgment, induces self-centered thinking and judgment in virtual environments and psychological distress, and contributes to raising depression. According to Moon et al. [29], these problems are significant and induce negative changes in daily and school life (e.g., learning, activities of daily life, and social interaction). Our finding of a positive relationship between smartphone overdependence and depression among high school students concurred with these studies above.

Various studies have previously verified the significant effect of smartphone overdependence on mental health such as obsessive behavior, anxiety, and depression [30]. Under these conditions, if individuals do not use their smartphones, abnormal symptoms in the autonomic nerve system appear, and psychological discomfort such as anger, irritability, and anxiety rises [1]. Most studies agree that depression is an important predictor of smartphone overdependence and the most important variable of mental health [30]. Moon et al. [29] reported that depression has a stronger relationship with smartphone overdependence than with other mental health factors and is a crucial factor determining the risk of smartphone addiction. Accordingly, this study's results have clinical significance. To decrease smartphone overdependence and depression, appropriate approaches and considerations are needed for high school students.

In this study, we found a negative effect of the quality of friendship on depression among high school students, indicating that if the quality of friendship decreases, the depression level increases. Various studies have previously reported that friendship is important for high school students. Cho and Kim [7] reported that friendship is an important activity to prepare for adulthood and form social roles and interpersonal skills. In addition, Kim et al. [8] reported that friendship plays an important role for students to experience social positions and status and learn methods to form appropriate interpersonal relationships as well as form self-identity, confidence, and values. However, problems with friendships in this period increase emotional instability, hamper the formation of appropriate values and self-identity, and increase negative emotions such as feelings of uncertainty and disconnection [9].

A decrease in the quality of friendship directly limits social interaction and raises psychological distress. Thus, when the performance of social roles conflicts, the depression level increases significantly [8]. Buck and Dix [31] reported that among adolescents, friendship quality mediates the relationship between inhibition and depression symptoms and that inhibition increases conflict, while conflict decreases support and positive affect among friends. Thus, the quality of friendship induces loneliness and social dissatisfaction and can lower mental health. Nangle et al. [32] also reported that the quality of friendship is significantly related to depression mediated by loneliness. According to these studies, such problems lead to adaptation challenges in daily and school life among high school students and lower academic achievement. Thus, to decrease the depression level and improve the quality of friendship among high school students, appropriate measures should be prepared and applied.

In addition, the results of the multiple linear regression analysis showed that the quality of friendship has a greater effect on the depression level than does smartphone overdependence. Friendship among high school students is important for their psychological and social development and helps them construct their identity [33]. In particular, friendship quality determines their success in social relationships and affects their psychological adjustment and social competence [34]. Thus, high school students who have close, stable, and supporting friendships tend to experience fewer interpersonal conflicts and a lower level of depression [33]. The use of smartphones enables wider interpersonal relations and better relationship-building with friends using various apps and mobile content [35]. Indeed, smartphone use plays a positive role in maintaining comfortable relations and making friends with people with common interests [33].

However, Matsuda [36] reported that such selective friendships (i.e., maintaining only personally comfortable relations and making friends with those with common interests) makes people's friendships close and suggests a potential risk of closed interpersonal relations. In addition, Devitt and Roker [37] stated that during smartphone use, most people fail to understand each other because of the use of non-verbal elements such as gestures and facial expressions. These problems induce interpersonal conflicts. When communicating with others using a smartphone, about 28% of the surveyed respondents in Kamibeppu and Sugiura's [35] study experienced their message being misunderstood and about 48% felt insecure when their messages were not answered, suggesting that relatively many people feel emotional instability during communication. Thus, to analyze the causal relationships and mediating effects among smartphone overdependence and the quality of friendship, causal and path analyses should be conducted.

The study's limitations were as follows. The purpose of this study was to analyze the effects of smartphone overdependence and the quality of friendship on depression among high school students. The correlation analysis showed statistically significant relationships among all the variables. However, according to the multiple linear regression analysis, the effects were confirmed only between smartphone overdependence and the quality of friendship/depression. Thus, follow-up studies should aim to verify the effects of smartphone overdependence and the quality of friendship and confirmatory factor analysis and path analysis should be conducted to analyze the effects among the variables. Moreover, this study did not analyze the sub-factors of smartphone overdependence. Thus, it did not verify the relationships and effects of the sub-factors of smartphone overdependence. Follow-up studies could aim to examine the relationships and effects of the sub-factors of smartphone overdependence on the variables. Lastly, this study did not compare groups, as it had a single-group study design. Therefore, a comparative analysis study with other groups is necessary in the future.

## 5. Conclusion

This study analyzed the effects of smartphone overdependence and the quality of friendship on depression among high school students. We found a positive correlation between smartphone overdependence and the depression level, indicating that an increase in smartphone overdependence raises the level of depression. In addition, we found a negative correlation between the quality of friendship and depression, indicating that a decrease in the quality of friendship raises the level of depression. The effect of the quality of friendship on depression was higher than that of smartphone overdependence on depression. Thus, to decrease the depression level, smartphone overdependence and the quality of friendship should be managed properly among high school students. Further, the causal relationships and mediating effects between smartphone overdependence and the quality of friendship should be analyzed more in detail.

## Figures and Tables

**Table 1:** General characteristics of the subjects (*n* = 121).

Age (years)	Sex (*n*, %)		Grade (*n*, %)	
16.69 ± .46	Male	Female	Second grade	121 (100)
	70 (57.85)	51 (42.15)		

**Table 2:** Results of the analysis of each variable.

Variable	Mean	S.D.	Range	Skewness	Kurtosis
Smartphone overdependence (points)	20.36	5.91	29.00 (10–39)	.225	.045
Depression (points)	4.22	5.20	27.00 (0–27)	2.275	6.591
Quality of friendship (points)	79.33	10.99	44.00 (61–105)	.109	-.186

∗∗*p* < .01.

**Table 3:** Results of the correlation analysis among the variables.

Variable	1	2	3
1. Smartphone overdependence (points)	1		
2, depression (points)	.343∗∗	1	
3. Quality of friendship (points)	-.203∗	-.600∗∗	1

∗∗*p* < .01, ∗*p* < .05.

**Table 4:** Results of the multiple regression analysis among the variables.

Variable	Coef.	S.E.	*t*
Smartphone overdependence	.203∗∗	.063	3.20
Quality of friendship	-.261∗∗∗	.034	-7.66
Constant	20.817∗∗∗	3.249	6.41
*R* ^2^	.411		
Adj. *R*^2^	.401		
*F* (2,118)	41.12∗∗∗		
*N*	121		

∗∗∗*p* < .001, ∗∗*p* < .01.

**Table 5:** Results of White's test.

Item	Chi^2^	Df	*p*
Heteroscedasticity	34.90	5	.00∗∗∗
Skewness	18.87	2	.00∗∗∗
Kurtosis	3,12	1	.08

∗∗∗*p* < .001.

**Table 6:** Results of the multiple regression analysis with RDWLS among the variables.

Variable	Coef.	S.E.	*t*
Smartphone overdependence	.203∗	.087	2.34
Quality of friendship	-.261∗∗∗	.042	-6.23
Constant	20.817∗∗∗	3.644	5.71
*R* ^2^	.411		
Adj. *R*^2^	.402		
*F* (2,118)	20.39∗∗∗		
*N*	121		

∗∗∗*p* < .001, ∗*p* < .05.

## Data Availability

The datasets generated and/or analyzed during this study are from the high school students. Thus, after obtaining the subjects' permission of this study subjects, they are available from the corresponding author on reasonable request.

## References

[1] Hwang K. H., Yoo Y. S., Cho O. H. (2012). Smartphone overuse and upper extremity pain, anxiety, depression, and interpersonal relationships among college students. *The Journal of the Korea Contents Association*.

[2] Park J. M., Kang M. K. (2019). Smartphone addiction and uses of high school students. *Asia-Pacific Journal of Multimedia Services Convergent with Art, Humanities, and Sociology*.

[3] Oh S. T., Kim J. U., Park S. C. (2015). The effects of technostress and work connectivity after work hours on job satisfaction: focusing on a mediating role or work-life conflicts. *Journal of Information Technology Applications & Management*.

[4] Kim T. J., Kim S. Y. (2015). Smartphone use pattern and academic achievement. *Journal of Government Administration*.

[5] Bae S. M. (2018). Influence of smartphone usage types and excessive expectation for smartphone on adolescents’ smartphone overdependence. *Informatization Policy*.

[6] National Information Society Agency (NIA) (2020). *Survey about smartphone overdependence in 2020*.

[7] Cho S. Y., Kim K. C. (2014). The effects of career identity, career decision level and career maturity for middle-high school students. *Korean Journal of Youth Studies*.

[8] Kim H. S., Choi Y. H., Yoo S. J. (2010). The study on the relations among ego-identity, stress, and internet addiction in high school students. *Journal of Korean Academy of Psychiatric and Mental Health Nursing*.

[9] Lee M. S., Kim K. Y., Ko K. J. (2003). A study on the related factors with internet addiction of the 11^th^ grade students in an urban area. *Journal of Preventive Medicine and Public Health*.

[10] Kim Y. O., Shim M. S. (2015). Cognitive functions, instrumental activities of daily living, depression and quality of life in the elderly with mild cognitive impairment. *Journal of Korean Public Health Nursing*.

[11] Kim Y. H., Lee C. H. (2017). The relationship between smartphone addiction and academic engagement of specialized high school students. *The Korean Journal of Technology Education*.

[12] Jo E. J., Kim Y. J., Kwon E. B., Lee D. H. (2020). Effect of smart-phone addiction on school adjustment of high school students: focused on mediating effect of psychological distress. *The Journal of the Korea Contents Association*.

[13] Kim D. S. (2018). The structural relationship among smartphone dependency, internet cognitive failure, peer relationship, academic stress and happiness of high school students. *The Korea Journal of Youth Counseling*.

[14] Oh J. (2015). The effects of high school students’ smart phone addiction on impulsivity, stress, self-efficacy, and self-control. *Journal of Fisheries and Marine Sciences Education*.

[15] Woo J. J., Kwak E. M., Lee H. J. (2018). The convergence study of smartphone overuse on cyberbullying: focusing on mediating effects of aggression. *Journal of the Korea Convergence Society*.

[16] Choi H. S., Choi J. H., Park K. H. (2007). Standardization of the Korean version of patient health questionnaire-9 as a screening instrument for major depression disorder. *Korean Journal of Family Medicine*.

[17] Kroenke K., Spitzer R. L., Williams J. B. (2001). The PHQ-9. *Journal of General Internal Medicine*.

[18] Parker J. G., Asher S. R. (1993). Friendship and friendship quality in middle childhood: links with peer group acceptance and feelings of loneliness and social dissatisfaction. *Developmental Psychology*.

[19] Kim E. J. (2010). Validation of a Korean version of the friendship quality questionnaire. *Korean Journal of Youth Studies*.

[20] Kim M. H., Oh I. S. (2019). A study on the relationship between parental overprotection and college student burnout: the moderated mediating effect of ego-resiliency and friendship quality. *Journal of Educational Innovation Research*.

[21] West S. G., Finch J. F., Curran P. J., Hoyle R. G. (1995). Structural equation models with non-normal variables: problems and remedies. *Structural Equation Modeling: Concepts, Issues, and Applications*.

[22] Bertozzi L., Negrini S., Agosto D. (2021). Posture and time spent using a smartphone are not correlated with neck pain and disability in young adults: a cross-sectional study. *Journal of Bodywork and Movement Therapies*.

[23] Lim L., Chang S. H., Lee J., Kim K. (2017). Effects of smartphone texting on the visual perception and dynamic walking stability. *Journal of Exercise Rehabilitation*.

[24] Berolo S., Wells R. P., Amick B. C. (2011). Musculoskeletal symptoms among mobile hand-held device users and their relationship to device use: a preliminary study in a Canadian university population. *Applied Ergonomics*.

[25] Lee H. G., Son J. H. (2020). The mediating effect of interpersonal relationship problems on the association of depression and internet smartphone addiction in high school boys. *The Korea Journal of Youth Counseling*.

[26] Kim S. H., Jeong I. S. (2014). Agreement between smartphone addiction and perceived smartphone among adolescents. *The Journal of Korean Society for School & Community Health Education*.

[27] Röösli M., Frei P., Mohler E., Hug K. (2010). Systematic review on the health effects of exposure to radiofrequency electromagnetic fields from mobile phone base stations. *Bulletin of the World Health Organization*.

[28] Shim M. Y., Lee D. N., Kim E. H. (2016). A study on influential relations between stress and smartphone addiction among college students: with a focus on the mediating effects of depression and self-efficacy. *Journal of the Korea Academia-Industrial Cooperation Society*.

[29] Moon J. H., Song E. S., Seong H. Y. (2019). Investigation of self-rated health and happiness, physical activity, and mental health by smartphone overuse using Korea youth risk behavior web-based survey 2017. *Journal of the Korea Entertainment Industry Association*.

[30] Lee H. G. (2009). xploratory the predicting variables of the addictive mobile phone use of teenage comparison 20 and 30 ages. *Korean Journal of Youth Studies*.

[31] Buck K. A., Dix T. (2012). Can developmental changes in inhibition and peer relationships explain why depressive symptoms increase in early adolescence?. *Journal Youth Adolescence*.

[32] Nangle D. W., Erdley C. A., Newman J. E., Mason C. A., Carpenter E. M. (2003). Popularity, friendship quantity, and friendship quality: interactive influences on children’s loneliness and depression. *Journal of Clinical Child & Adolescent Psychology*.

[33] Kharimah U. N., Prasetyawati W., Sary M. P. (2018). Association between friendship quality and depression among high school students in Jakarta. *Advances in Social Science, Education and Humanities Research*.

[34] Berndt T. J. (2002). Friendship quality and social development. *American Psychological Society*.

[35] Kamibeppu K., Sugiura H. (2005). Impact of the mobile phone on junior high-school students' friendships in the Tokyo metropolitan area. *Cyberpsychology & Behavior*.

[36] Matsuda M. (2000). Friendship of young people and their usage of mobile phones: from the view of superficial relation to selective relation. *Shakai Jouhougaku Kenkyuu*.

[37] Devitt K., Roker D. (2009). The role of mobile phones in family communication. *Children & Society*.

